This article has been retracted.

# Relationship between Severity of Lumbar Spinal Stenosis and Ligamentum Flavum Hypertrophy and Serum Inflammatory Factors

**DOI:** 10.1155/2022/8799240

**Published:** 2022-10-12

**Authors:** Nina He, Wenbin Qi, Yongli Zhao, Xiaojun Wang

**Affiliations:** Department of Rehabilitation Physiotherapy, Shandong University Qilu Hospital (Qingdao), Qingdao, Shandong 266000, China

## Abstract

**Objective:**

This study is aimed at investigating the correlation between lumbar spinal stenosis (LSS) severity, ligamentum flavum hypertrophy, and the upregulation of inflammatory markers.

**Methods:**

From March 2019 and May 2022, eighty-five inpatients with LSS were enlisted as the study's research group, while sixty-five patients hospitalized for lumbar intervertebral disc herniation over the same time period served as the study's control group. Moreover, mild, moderate, and severe subgroups of patients were created within the research population based on their LSS severity. The ligamentum flavum thickness and the positive expression rates of TNF-*α*, TGF-*β*1, and IL-1*α* were compared between the study group and the control group. The levels of TNF-*α*, TGF-*β*1, and IL-1*α* that were found to be positively expressed were compared between the mild, moderate, and severe groups. Patients with LSS had their ligamentum flavum thickness and their positive expression rates of TNF-*α*, TGF-*β*1, and IL-1*α* analyzed using Spearman correlation analysis. We evaluated the diagnostic utility of the positive expression rates of IL-*α*1, TGF-*β*1, and TNF-*α* and ligamentum flavum thickness in distinguishing the severity of LSS using a receiver operating characteristic (ROC) curve.

**Results:**

The rates of both lower limb pain (40.00%) and intermittent claudication (80.00%) in the LSS group were higher than those in the lumbar disc herniation group (15.38%, 12.31%), with statistical significance (*P* < 0.05). However, no substantial disparity was observed in left lower limb pain, right lower limb pain, low back pain, lower limb sensation, muscle strength, and reflex abnormalities between the two groups (*P* > 0.05). Positive expressions of TGF-*β*1, TNF-*α*, and IL-1*α* and thicker ligamentum flavum were more prevalent in the LSS group than in the lumbar intervertebral disc herniation group. All indexes were significantly (*P* < 0.05) higher in the moderate stenosis group than in the severe stenosis group. Additionally, the thickness of the ligamentum flavum and the positive expression rates of TNF-*α*, TGF-*β*1, and IL-1*α* were higher in the mild and moderate stenosis groups than in the severe stenosis group. The expression levels of TNF-*α*, TGF-*β*1, and IL-1*α* were favorably linked with ligamentum flavum thickness (*P* < 0.05). ROC curve analysis showed that the thickness of ligamentum flavum, the expression of IL-1*α*, the expression of TGF-*β*1, and the expression of TNF-*α* could effectively diagnose mild, moderate, and severe LSS (*P* < 0.05).

**Conclusion:**

Ligamentum flavum hypertrophy and positive expression rates of IL-1*α*, TGF-*β*1, and TNF-*α* are closely linked to LSS, which can effectively identify mild, moderate, and severe LSS.

## 1. Introduction

Lumbar spinal stenosis (LSS) can cause lumbago and leg pain or lower extremity motor dysfunction in middle-aged and elderly people. The pathogenesis is mainly intervertebral disc bulge, protrusion or degenerative calcification, vertebral joint hyperplasia and ossification, ligamentum flavum hypertrophy, and calcification, which can lead to stenosis of the spinal canal, lateral recess, nerve root canal, or foramina, thus causing a series of symptoms such as compression of cauda equina nerve, blood vessels, and nerve roots in the dural sac or inflammatory reactions [1, 2]. Anatomically, there are three distinct forms of LSS: lateral foraminal, recess, and central canal stenosis. Degeneration of the facet joints, ligamentum flavum and intervertebral disc are the primary anatomical factors in central stenosis. The degeneration of the intervertebral disc often has a high degree of loss, and the hypertrophic ligamentum flavum can form space behind both sides of the spinal canal, further aggravating the central stenosis [3–5]. Lateral recess stenosis is mostly caused by the proliferation of osteophytes on the medial side of the superior articular process, which is related to disc herniation and inflammatory response of the articular process. Foraminal stenosis is caused by osteophytes above the articular process and is associated with disc degeneration. Various inflammatory factors and increased load stress can lead to ligamentum flavum injury, and the repair process is accompanied by ligament fibrosis and collagen fiber hyperplasia, resulting in ligamentum flavum hypertrophy [6–8]. The goal of this research was to examine the connection between degenerative hypertrophy of the ligamentum flavum and the development of LSS and an inflammatory response, so as to further improve the prevention, diagnosis, and treatment of LSS and provide theoretical support for clinical treatment of LSS.

## 2. Materials and Methods

### 2.1. General Information

The selection included 85 LSS patients who received care at our facility between March 2019 and May 2022, and 65 patients with lumbar intervertebral disc herniation who were hospitalized during the same period were selected. There were 51 men and 34 females in the LSS group, with ages ranging from 40 to 75 (56.96 ± 7.05 years) and disease durations averaging 29.22 ± 9.46 months (range = 10 to 55). There were 40 men and 25 females in the lumbar disc herniation cohort; the age range was from 42 to 72 years old, with a mean age of 55.97 ± 7.38 years; the duration of disease was from 6 to 45 months, with a mean of 30.74 ± 8.01 months. Overall, there was comparable difference between the two groups' data (*P* > 0.05). Eventually, MRI and CT scans were performed on every patient. Patients with LSS were categorized into those with mild stenosis (23 cases), moderate stenosis (45 cases), and severe stenosis (17 cases), depending on the number of stenotic segments in their arteries. The hospital's ethics board gave its stamp of approval to this research. Inclusion criteria include ① patients diagnosed with LSS or lumbar disc herniation by imaging examination, ② central stenosis, ③ complete lumbar spine imaging data, and ④ all patients who voluntarily participated in this study. Exclusion criteria include ① those who have suffered a spinal fracture or spinal cord damage, ② patients with developmental lumbar spinal stenosis, ③ patients complicated with spinal tumor, spinal deformity, and other spinal diseases, ④ patients with osteoarticular tuberculosis, osteomyelitis, and severe senile osteoporosis, and ⑤ patients with severe organ dysfunction.

### 2.2. Methods

① Thickness measurement of ligamentum flavum: all patients underwent CT scanning at different lesion segments (L3/L4, L4/L5, and L5/S1). The oblique diameter of the spinal canal was measured and compared to the thickness of the ligamentum flavum of both joint capsules to determine the disc height ratio at the superior vertebral arch notch. ② Lamina ligamentum flavum was removed during posterior spinal canal and lateral recess decompression, rinsed in 0.9% sodium chloride solution, fixed in 4.0% paraformaldehyde, embedded in paraffin, and cut into 5-8 pieces for immunohistochemistry staining. Immunohistochemical staining sections of transforming growth factor- (TGF-) *β*1, tumor necrosis factor- (TNF-) *α*, and interleukin- (IL-) 1*α* in the two groups were observed with Olympus light microscope (Japan) by two-person double-blind method. The sections of each group were placed under the same intensity light, and 5 visual fields were randomly selected from each section under a high-power microscope (×40). Judgment of immunohistochemical results: if there were brown or dark brown particles in the cytoplasm or membrane of the ligamentum flavum tissue and the staining intensity was higher than the background nonspecific staining, the cells were considered positive. If the nucleus was stained blue and there was no brown-yellow reactant in the membrane or cytoplasm, the cells were considered negative. Five complete and nonoverlapping high magnification fields were selected at the tissue edge of ligamentum flavum in each section, and the expression rate of positive cells in each field was measured. The average expression rate of 5 fields was taken as the final measurement value. Positive cell expression rate: 0 indicates no expression (-); <25% indicates slight expression (+); ≥25% indicates obvious expression (++). The expression degree and positive expression rate of three inflammatory factors including TGF-*β*1, TNF-*α*, and IL-1*α* in the ligamentum flavum of the two groups were compared.

### 2.3. Observation Indicators

The indicators are as follows: ① comparison of ligamentum flavum thickness and expression quantity of TGF-*β*1, TNF-*α*, and IL-1*α* between the LSS group and the lumbar disc herniation group; ② comparison of ligamentum flavum thickness and expression quantity of TGF-*β*1, TNF-*α*, and IL-1*α* in mild, moderate, and severe stenosis groups; ③ correlation analysis between the severity of LSS and the expression quantity of TGF-*β*1, TNF-*α*, and IL-1*α* and the ligamentum flavum thickness; ④ the ROC curve analysis of TGF-*β*1, TNF-*α*, and IL-1*α* and ligamentum flavum thickness in differentiating the severity of LSS.

### 2.4. Statistical Methods

Data for this study were entered into an Excel spreadsheet by two researchers working independently of one another and then analyzed and processed using SPSS 24.0. In this study, we used a mean ± SD (*x* ± *s*) format for our measurement data. When the data follows a normal distribution with consistent variance, the *t*-test is used. *n* and % were utilized to characterize the count data, and the chi-square test was performed to compare the two groups. All were two-sided tests. The relationship between the thickness of the ligamentum flavum and the levels of TGF-*β*1, TNF-*α*, and IL-1*α* in individuals with LSS was examined using Spearman correlation analysis. *P* < 0.05 was regarded as a statistically significant difference when analyzing the diagnostic value of ligamentum flavum thickness and the positive expression rates of TGF-*β*1, TNF-*α*, and IL-1*α* in determining the degree of LSS using the receiver operating characteristic (ROC) curve.

## 3. Results

### 3.1. The Signs and Clinical Symptom Comparison between the Two Groups

Both lower extremity pain (40.00%) and intermittent claudication (80.00%) were more prevalent in the LSS group than in the lumbar disc herniation group, with a statistically significant difference (*P* < 0.05) between the two groups. Left lower extremity pain, right lower extremity pain, low back pain, lower extremity sensation, muscle strength, and reflex abnormalities were all similar across the two groups (*P* > 0.05). See Table 1.

### 3.2. Comparison of Ligamentum Flavum Thickness and Positive Expression Rates of TGF-*β*1, TNF-*α*, and IL-1*α* between the Two Groups

The ligamentum flavum thickness in the LSS group was greater than that in the lumbar intervertebral disc herniation group. There was a statistically significant (*P* < 0.05) increase in the TGF-*β*1, TNF-*α*, and IL-1*α* positive expression when compared to the group with lumbar intervertebral disc herniation (Table 2).

### 3.3. Comparison of Ligamentum Flavum Thickness and TGF-*β*1, TNF-*α*, and IL-1*α* Positive Expression Rate among Three Subgroups

There were significant differences in the ligamentum flavum thickness and the TGF-*β*1, TNF-*α*, and IL-1*α* positive expression among the three subgroups (*P* < 0.05). There were statistically significant (*P* < 0.05) increases in ligamentum flavum thickness, TGF-*β*1, TNF-*α*, and IL-1*α* positive expression, and each index in the moderate stenosis group compared to the severe stenosis group, as shown in Figures 1 and 2 and Table 3.

### 3.4. Correlation Analysis between Ligamentum Flavum Thickness and TGF-*β*1, TNF-*α*, and IL-1*α* Expression

The ligamentum flavum thickness was positively correlated with the expressions of IL-1*α*, TGF-*β*1, and TNF-*α* (*P* < 0.05). See Figure 3.

### 3.5. ROC Curve Analysis of Expression Quantity of TNF-*α*, TGF-*β*1, and IL-1*α* and Ligamentum Flavum Thickness in Differentiating the Severity of LSS

ROC curve analysis showed that the ligamentum flavum thickness and TGF-*β*1, TNF-*α*, and IL-1*α* expression could effectively diagnose mild, moderate, and severe LSS (*P* < 0.05). The AUC values of ligamentum flavum thickness and expression quantity of TNF-*α*, TGF-*β*1, and IL-1*α* in the identification of mild to moderate LSS were 0.986, 0.825, 0.765, and 0.976, respectively, and the cut-off values were 4.67, 89.18, 73.93, and 42.14, respectively. The AUC values of ligamentum flavum thickness and expression quantity of TNF-*α*, TGF-*β*1, and IL-1*α* in the identification of moderate to severe LSS were 0.835, 0.742, 0.890, and 0.891, and the cut-off values were 6.62, 94.66, 80.89, and 50.55, respectively. See Tables 4 and Tables 5 and Figures 4 and 5.

## 4. Discussion

Hypertrophy and ligamentum flavum hypertrophy may cause a narrowing of the spinal canal (coronal diameter), as well as hyperplasia and cohesiveness of the bilateral facet joints and the superior facet joints, all of which increase the chances of LSS [9–11]. Patients with mild LSS should be treated with rest, drugs, and relevant symptomatic treatment. Patients with severe LSS accompanied by intractable pain and ineffective nonsurgical treatment should be treated with surgery. The degenerated and herniated intervertebral discs and facet joints act on the ligamentum flavum by releasing inflammatory factors, causing ligamentum flavum hypertrophy [12, 13]. IL-1*α* can promote the formation of inflammation and cause pain. IL-1*α* is a predisposed factor for the thickening and ossification of ligamentum flavum, which can affect ligamentum flavum by stimulating nerves, degrading collagen, and mediating cycloxygenase-2 metalloproteinase inhibitors. The positive expression rate of IL-1*α* in the LSS group was substantially greater than that in the control group in this research, which may be related to chronic mechanical effects and increased pain in patients with LSS, and pain is caused by stimulation of nerve fibers. The ligamentum flavum was thicker and fibrotic in the LSS group, with fibroblasts serving as the predominant cell type, so the positive expression of IL-1*α* was increased. According to relevant studies, IL-1*α* is highly expressed in the intervertebral disc and lumbar facet joint and patients with lumbar stenosis tend to have a more active ligamentum flavum, and this activity is positively connected with lumbar region and leg pain [14, 15]. Hypertrophy of the ligamentum flavum in the lumbar spine causes a loss of elasticity and an increase in collagen fibers [16, 17]. It has been suggested that TGF-*β*1 is closely related to fibroblast proliferation [18, 19]. TGF-*β*1 can change the growth characteristics of fibrocytes and reduce the contact inhibition effect in the process of fibrocyte growth. It can not only promote cell proliferation but also promote the synthesis of extracellular matrix. Since TGF-*β*1 can cause a variety of tissue hypertrophy, which is closely related to a variety of fibrotic diseases, the mechanism of TGF-*β*1 promoting ligament flavum hypertrophy lies in inducing fibroblast differentiation into myofibroblasts, which can promote the fibrosis of ligament flavum tissue by promoting the production of type I and III collagen [20]. Therefore, the main role of TGF-*β*1 in inducing ligamentum flavum hypertrophy is to promote the proliferation and differentiation of fibroblasts and the formation of collagen fibers. TNF-*α* mainly affects the metabolism of collagen fibers in the ligamentum flavum matrix. TNF-*α* is an inflammatory factor secreted by macrophages, which is an initiating factor of inflammatory cascade reaction and can reflect the severity of inflammation [21, 22]. According to relevant studies, TNF-*α* content is closely related to the effect of macrophage migration inhibitory factor (MIF), which is an upstream factor of TNF-*α* and can promote the expression of TNF-*α* in fibroblasts and stroma. In addition, MIF can indirectly promote the expression of TNF-*α* by inhibiting the migration of macrophages [23, 24]. In addition, ligamentum flavum hypertrophy may be caused by TNF-*α* due to its ability to stimulate the production of downstream metalloproteinases through positive feedback. Ligamentum flavum has both type I and type III collagen fibers. Hypertrophy of the ligamentum flavum is associated with TNF-*α* because TNF-*α* may increase the production of type III collagen.

In this study, in patients with LSS, the ligamentum flavum was thicker than in those with lumbar disc herniation, and the LSS group also had higher levels of TGF-*β*1, TNF-*α*, and IL-1*α* positive expression. Each indicator was greater in the moderate stenosis group than the severe stenosis group, and the differences between the groups were statistically significant (*P* < 0.05). Positive expression rates of TNF-*α*, TGF-*β*1, and IL-1*α* increased with increasing stenosis severity, and the findings demonstrated that these cytokines were strongly expressed in the LSS group. The degree of LSS was correlated with an increase in ligamentum flavum thickness, which was considerably greater in the LSS group than in the lumbar disc herniation group. Clinical studies have shown that corticosteroids and nonsteroidal analgesic and anti-inflammatory drug COX-2 inhibitors can relieve clinical symptoms by inhibiting inflammatory response, and patients with LSS often have ligamentum flavum hypertrophy. In this work, we found that LSS was closely linked with the TGF-*β*1, TNF-*α*, and IL-1*α* positive expression rate as assessed by Spearman's correlation analysis (*P* < 0.05). Previous research has shown that TNF-*α* and IL-1*α* are both substantially expressed in the intervertebral discs, lumbar facet joints, and ligamentum flavum of individuals with LSS and that this expression is connected with neurological dysfunction and lumbar and leg pain [25, 26]. IL-1*α* can enhance the synthesis of pain mediators prostaglandin and 5-hydroxytryptamine. Prostaglandin E2 is an important transmitter of inflammatory response, which can enhance the sensitivity of nerve terminal receptors, thus enhancing the pain effect. IL-1*α* induces nerve root pain through mediating other inflammatory mediators, eventually leading to lumbar and leg pain. TNF-*α* can induce inflammatory reactions such as endoneurial edema, decreased blood flow, intravascular coagulation, and medulla decomposition, which can play a role in the regulation of nerve root sensitivity and cause lumbar and leg pain. Lumbar and leg pain is the main symptom of LSS, which can also explain that the expression of inflammatory factors increases with the degree of LSS.

ROC curve analysis results of this study showed that the thickness of ligamentum flavum and the expression quantity of TNF-*α*, TGF-*β*1, and IL-1*α* could effectively diagnose mild, moderate, and severe LSS (*P* < 0.05). The AUC values of ligamentum flavum thickness and expression quantity of TNF-*α*, TGF-*β*1, and IL-1*α* in identifying mild to moderate LSS were 0.986, 0.825, 0.765, and 0.976, respectively, and the cut-off values were 4.67, 89.18, 73.93, and 42.14, respectively. The AUC values of ligamentum flavum thickness and expression quantity of IL-1*α*, TGF-*β*1, and TNF-*α* in identifying moderate to severe LSS were 0.835, 0.742, 0.890, and 0.891, respectively, and the cut-off values were 6.62, 94.66, 80.89, and 50.55, respectively. For patients with mild LSS, rest, medication, and relevant symptomatic treatment are required, while surgery may be required for patients with moderate and severe LSS. Early identification of patients after admission is beneficial to quickly determine the treatment plan, and appropriate treatment plan can promote the rational utilization of medical resources and improve the prognosis of patients, suggesting that the thickness of ligamentum flavum can be measured in patients with LSS after admission. In this study, the TGF-*β*1, TNF-*α*, and IL-1*α* positive expression rate was determined by postoperative immunohistochemistry, which can reveal the expression patterns of inflammatory factors in patients with LSS.

In conclusion, the severity of LSS is closely correlated with ligamentum flavum hypertrophy and the expression quantity of TNF-*α*, TGF-*β*1, and IL-1*α*. Ligamentum flavum hypertrophy and the TGF-*β*1, TNF-*α*, and IL-1*α* positive expression rate can effectively distinguish the LSS severity.

## Figures and Tables

**Figure 1:** Comparison of ligamentum flavum thickness among three subgroups.

**Figure 2:** Comparison of positive expression rates of TNF-*α*, TGF-*β*1, and IL-1*α* among three subgroups.

**Figure 3:** Correlation between ligamentum flavum thickness and expression quantity of IL-1*α*, TGF-*β*1, and TNF-*α*.

**Figure 4:** ROC curve analysis of IL-1*α*, TGF-*β*1, and TNF-*α* expression quantity and ligamentum flavum thickness in differentiating mild to moderate LSS.

**Figure 5:** ROC curve analysis of IL-1*α*, TGF-*β*1, and TNF-*α* expression quantity and ligamentum flavum thickness in differentiating moderate to severe LSS.

**Table 1:** Comparison of clinical symptoms and signs between the two groups [*n* (%)].

Group	Left lower extremity pain	Right lower extremity pain	Both lower extremity pain	Low back pain	Lower extremity sensation, muscle strength, and reflex abnormalities	Intermittent claudication
LSS group (*n* = 85)	24 (28.24)	27 (31.76)	34 (40.00)	68 (80.00)	78 (91.76)	68 (80.00)
Lumbar disc herniation group (*n* = 65)	23 (35.38)	23 (35.38)	10 (15.38)	55 (84.62)	62 (95.38)	8 (12.31)
*χ* ^2^ value	0.875	0.217	10.767	0.532	0.776	67.524
*P* value	0.350	0.641	0.001	0.466	0.378	<0.001

**Table 2:** Comparison of ligamentum flavum thickness and TGF-*β*1, TNF-*α*, and IL-1*α* positive expression rate between the two groups (^−^*x* ± *s*).

Group	Ligamentum flavum thickness (mm)	IL-1*α* (%)	TGF-*β*1 (%)	TNF-*α* (%)
LSS group (*n* = 85)	5.55 ± 1.51	90.66 ± 8.31	75.14 ± 9.03	45.37 ± 7.15
Lumbar disc herniation group (*n* = 65)	2.51 ± 0.70	12.97 ± 3.78	46.20 ± 6.02	8.53 ± 3.03
*t* value	16.408	76.528	23.488	42.776
*P* value	<0.001	<0.001	<0.001	<0.001

**Table 3:** Comparison of ligamentum flavum thickness and positive expression rates of TNF-*α*, TGF-*β*1, and IL-1*α* among three subgroups (^−^*x* ± *s*).

Group	Ligamentum flavum thickness (mm)	IL-1*α* (%)	TGF-*β*1 (%)	TNF-*α* (%)
Mild stenosis group (*n* = 23)	3.53 ± 0.51	83.63 ± 4.87	67.45 ± 7.54	36.95 ± 4.19
Moderate stenosis group (*n* = 45)	5.97 ± 0.76^a^	91.43 ± 7.16^a^	75.42 ± 7.41^a^	46.47 ± 3.91^a^
Severe stenosis group (*n* = 17)	7.17 ± 0.90^ab^	98.13 ± 7.53^ab^	84.77 ± 3.96^ab^	53.85 ± 4.49^ab^
*F* value	135.287	23.500	30.770	86.277
*P* value	<0.001	<0.001	<0.001	<0.001

Note: ^a^*P* < 0.05 when compared with the mild stenosis group; ^b^*P* < 0.05 when compared with the moderate stenosis group.

**Table 4:** ROC curve analysis of expression quantity of IL-1*α*, TGF-*β*1, and TNF-*α* and ligamentum flavum thickness in differentiating mild to moderate LSS.

	AUC	*P* value	Cut-off value	95% CI
Ligamentum flavum thickness	0.986	<0.001	4.67	0.968-1.000
IL-1*α* expression quantity	0.825	<0.001	89.18	0.729-0.921
TGF-*β*1expression quantity	0.765	<0.001	73.93	0.646-0.884
TNF-*α* expression quantity	0.976	<0.001	42.14	0.947-1.000

**Table 5:** ROC curve analysis of expression quantity of IL-1*α*, TGF-*β*1, and TNF-*α* and ligamentum flavum thickness in differentiating moderate to severe LSS.

	AUC	*P* value	Cut-off value	95% CI
Ligamentum flavum thickness	0.835	<0.001	6.62	0.716-0.955
IL-1*α* expression quantity	0.742	0.003	94.66	0.598-0.887
TGF-*β*1 expression quantity	0.890	<0.001	80.89	0.809-0.971
TNF-*α* expression quantity	0.891	<0.001	50.55	0.807-0.975

## Data Availability

The labeled dataset used to support the findings of this study is available from the corresponding author upon request.
